# Regulation of T Cell Priming by Lymphoid Stroma

**DOI:** 10.1371/journal.pone.0026138

**Published:** 2011-11-14

**Authors:** Omar Khan, Mark Headley, Audrey Gerard, Wei Wei, Limin Liu, Matthew F. Krummel

**Affiliations:** 1 Department of Pathology, University of California San Francisco, San Francisco, California, United States of America; 2 Department of Microbiology and Immunology, University of California San Francisco, San Francisco, California, United States of America; Institut Pasteur, France

## Abstract

The priming of immune T cells by their interaction with dendritic cells (DCs) in lymph nodes (LN), one of the early events in productive adaptive immune responses, occurs on a scaffold of lymphoid stromal cells, which have largely been seen as support cells or sources of chemokines and homeostatic growth factors. Here we show that murine fibroblastic reticular cells (FRCs), isolated from LN of B6 mice, play a more direct role in the immune response by sensing and modulating T cell activation through their upregulation of inducible nitric oxide synthase (iNOS) in response to early T cell IFNγ production. Stromal iNOS, which only functions in very close proximity, attenuates responses to inflammatory DC immunization but not to other priming regimens and preferentially affects Th1 cells rather than Th2. The resultant nitric oxide production does not affect T cell-DC coupling or initial calcium signaling, but restricts homotypic T cell clustering, cell cycle progression, and proliferation. Stromal feedback inhibition thus provides basal attenuation of T cell responses, particularly those characterized by strong local inflammatory cues.

## Introduction

Naïve T cells are activated through surface presentation of peptide-MHC fragments by tissue-draining dendritic cells (DC). While the cell biology and dynamics of this isolated interaction have been extensively scrutinized[1]–[5], the interaction typically takes place against the background of lymphoid stroma, a collection of structural cells whose influence on the process has not been fully investigated.

Four cell types constitute the majority of stroma in secondary lymph nodes. Blood endothelial cells (BECs) are the structural cells that are assembled to form capillaries and high-endothelial venules (HEVs), structures T cells must traverse in order to enter the lymph node. Lymphatic endothelial cells (LECs), assemble the afferent and efferent lymphatic vessels, are largely contiguous with lymphatics themselves, and provide entry sites for dendritic cells arriving via lymph[6]. Within the lymph node, B cell zones are isolated and supported by follicular dendritic cells (FDCs) whereas fibroblastic reticular cells (FRCs) largely scaffold the T cell zone.

FRCs are thus the dominant stromal cell present at the site of T cell priming. These cells engulf reticular collagen fibers that weave throughout the T cell zone. The hollow core of the ensuing FRC network provides a conduit for soluble material to penetrate into the lymph node[7], [8]. FRCs also provide structure to the T cell zone and are hypothesized to act as ‘tracks’ for T cells to survey the contents of a node and on which chemokines may be immobilized for the purpose of guiding T cells[9]. They are also major sources of CCL19, CCL21 and IL-7, key factors guiding T cell motility and survival in the lymph node[10]. Finally, FRC appear to be direct targets of some viruses, resulting in viral modulation of CCL21 expression and possibly modulation of lymphoid homeostasis[11], [12]. In these various settings, FRC are seen largely to promote T cell survival and activation.

In this study, we investigated whether FRCs directly communicate with T cells activating in their midst and whether they are capable of providing specific feedback in the T cell priming process. We find that inclusion of FRC lines or freshly purified cells to T-DC priming cultures results in significant inhibition of activation. This inhibition does not rely on the FRC directly presenting antigens. FRC s are highly responsive to T cell-produced interferon gamma (IFNγ) and respond by upregulating their transcription of the *nos2* gene, encoding the enzyme inducible nitric oxide synthase (iNOS). The resulting nearby production of nitrite results in a block in T cell cell-cycle progression. We find that that iNOS inhibition during specific types of priming reactions in the lymph nodes plays a significant role in restricting T cell activation to immunization with inflammatory DC populations, consistent with a role in regulating the response. FRCs, prior and apart from this crosstalk, have no discernable effect on T cell priming at the level of signaling or expression of early activation markers. In sum, this places FRCs as regulators of T cell activation through direct communication with IFNγ producing T cells.

## Results

### Lymph node stromal cell populations inhibit naive T cell activation

In order to study the function of lymphoid stromal cells during T cell priming, we first established cell lines from the CD45 negative fraction of the LN, representing FRCs (“FRC.5”: gp38+, CD31−), LECs (“LEC.6”: gp38+CD31+) and BECs (“BEC.7”: gp38− CD31+) (**Fig 1a** **)**. These lines, once established, were passaged up to 10 times from each freeze and re-sorted between major freezes. These lines displayed distinct morphological features, consistent with their functions in situ; FRCs featuring very extended lamellopodia on plastic or glass surfaces and both LECs and BECs having elongated phenotypes with long extension (**Fig 1b**) and a high propensity to form side-by-side ‘bundles’ of cells in 2D cultures (not shown).

**Figure 1:** Inhibition of Initial T cell priming by Lymph node Stromal Populations. (**a**) Three cell lines were isolated representing FRC (FRC.5: CD31−/gp38+)), LEC (LEC.6: CD31+gp38+), and BEC (BEC.7: CD31+gp38−). (**b**) Contrast images of each line showing differences in morphology consistent with their in vivo function. (**c**) 10^5^ CFSE-labeled OTI T cells were incubated in 96-well round-bottom wells in the presence of 10^4^ BMDCs either unpulsed (NS) or pulsed (+SL8) with the indicated concentrations of SL8 peptides. 5×10^3^ stromal cells were added where indicated. Cells were analyzed by FACS after 48 hours. (**d**) CFSE proliferation assays were performed identically to (**a**) but included freshly purified gp38+CD31− FRC or an equal number of unfractionated total (including T cells, B cells, etc.) from collagenase digestion of lymph nodes. (**e**) Proliferation assays were performed identically to those in (**c,d**) but included mouse embryonic fibroblasts (MEF) or NIH-3T3 cells as 3^rd^ party cell types. All experiments are representative of at least 3 similar trials.

We subsequently tested the effects of each line, as a 5% cellular proportion, when co-cultured with a standard stimulation culture of naïve CD8 T cells, using monoclonal T cells derived from lymph nodes of OTI TCR transgenic mice mixed with in-vitro generated bone-marrow derived dendritic cells (BMDCs). T cells were labeled with CFSE to track cell division and, as shown in **Fig 1c** **,** in the absence of their cognate antigen, SIINFEKL (SL8), they did not divide, regardless of the presence of lymph node stromal lines. When BMDCs were pulsed with SIINFEKL peptide, T cells typically underwent multiple rounds of cell division within 48 hours. However, addition of FRC, LEC or BEC cell lines each resulted in nearly complete inhibition of the induced proliferation.

As T cell activation by DCs typically occurs in the T cell zone of lymph nodes, scaffolded by FRCs, we focused predominantly on these stromal cells and lines for subsequent studies. We first confirmed that freshly isolated gp38+CD31− CD45− FRCs were similarly inhibitory by assaying them in our T+DC stimulation cultures. In these assays, we compared FRC isolates to a similar number of total lymph node cells and found the FRCs (**Fig 1d**) again to be inhibitory for proliferation of CD8 T cells. To test for the specificity of inhibition, we also compared the FRC.5 line to mouse embryonic fibroblast lines (MEF) and fibroblasts (NIH-3T3) and found that whereas the latter lines also were modestly inhibitory for proliferation, the FRC.5 line consistently inhibited to a greater extent (**Fig 1e**). Given that the FRCs are present proximally in the LN during priming whereas BEC and LEC are not, we focused on the mechanism underlying their inhibition of the response.

### Inhibition of T cell activation by FRCs depends upon interferon gamma production during priming

We first sought to determine the magnitude of T cell inhibition and if it involved interactions between FRCs and DCs or was a direct effect upon T cells, regardless of DC presence. In **Fig 2a**, we added FRC.5 cells at varying levels to CFSE-loaded T cells and primed with a selection of stimuli. A 10% fraction of FRCs provided nearly complete blockade of T cell proliferation in response to BMDCs loaded with SL8, plate-bound anti-CD3 +/− soluble anti-CD28, or PMA plus ionomycin. However, when a smaller FRC concentration was used, there was little or no effect in some conditions but partial inhibition in the presence of αCD3 and αCD28. This implied that FRCs were not simply globally repressing responses but, rather, that they did so specifically in response to cues derived from the strength or type of activation of the T cells. We quantified this finding by a different criterion in **Fig 2b–c**. Here, we scored for the percentage of cells in the culture that were in or beyond the first division, and term this “% blasts”. By this criterion, which measures the degree to which cells are allowed to begin cycling, a greater distinction in the threshold of FRC-based inhibition emerged. We interpret from this that FRCs can very effectively inhibit the first cell division in some conditions (i.e. at 2.5% or more) such that very few cells progress to becoming ‘blasts’. In contrast, at the lower fractions (i.e. 1%), they inhibit this to a lesser extent but, for some priming conditions (e.g. BMDC), can prevent the maximal extent of cell cycling.

**Figure 2:** Regulation of T cell activation by LN Stromal cells via an IFNγ mediated and proximity-dependent mechanism. (**a–d**) CD8+ T cell proliferation under various stimuli. Cultures were incubated for 48 hours prior to analysis by flow cytometry. (**a**) CFSE dilution profiles of OTI T cells cultured with FRC.5 cells as well as either SL8 peptide-pulsed BMDCs (BMDC+SL8), plate-bound anti-CD3 (CD3), plate-bound anti-CD3 and soluble anti-CD28 (aCD3/aCD28), or soluble PMA and Ionomycin. (**b–d**) The percentage of blasting OTI cells are represented as the percentage of cells progressing past the first, non-proliferative, CFSE peak (% of Blasts). Cells were activated with various concentrations of FRC.5 under the following conditions: (**b**) activated with 10^4^ peptide-loaded BMDCs (**c**) plate-bound anti-CD3, plate-bound anti-CD3 and soluble anti-CD28, or soluble PMA and ionomycin and (**d**) various concentrations of total peptide-loaded BMDCs. (**e**) CFSE-based proliferation assay identical to that in (**a**) but also including soluble cytokines or cytokine-blocking antibodies that were added at the start of the assay as indicated in the legend. (**f**) Expression of the IFNγ receptor in FRC.5 or freshly *ex vivo* isolated FRC was analyzed by FACS and compared to reagent control. (**g**) Proliferation assay of SE-efluor670 labeled OTI cells. 6×10^5^ OTI cells and 6×10^4^ peptide-loaded BMDCs cultured in contact with 6×10^4^ FRC.5 cells (proximal) or separated from FRC.5 cells by a 0.4um transwell membrane (distal). All assays were repeated in a minimum of 2 and typically 4–6 independent trials and all conditions were assayed in triplicate. Error bars represent SD.

We used this same metric, while varying the number of BMDCs in the culture in order to test whether higher densities of DCs could overcome inhibition (**Fig 2d**). This revealed that the inhibition at the higher levels of FRCs could not be overcome with greater numbers of DCs, strongly suggesting that the inhibitory effect was not due to FRCs somehow confining DCs from T cells. The exclusion of such a mechanism was also supported by the ability of FRCs to inhibit T cell proliferation to the fully soluble PMA and Ionomycin stimulus (**Fig 2a** **and** **Fig 2c** **).**

Since it has been shown that distinct priming conditions result in differences in both the quantity and quality of cytokines produced by blasting T cells[13], [14], we sought to determine the effect of blocking select cytokines or adding them back to T+DC assays (**Fig 2e**). While we saw little effect of αIL4 or αIL-12 antibodies (data not shown), we found that addition of αIFN**γ** almost fully restored proliferation of T cells cultured with DCs in the presence of FRCs. Interleukin 2 nor αIL-2 had a significant effect on FRC-mediated inhibition of CFSE dilution. This implied that, at a strength of stimulation resulting in strong IFNγ secretion, FRCs were licensed to inhibit the T cell response. That FRC might be responsive to IFNγ was also supported by their robust expression of the IFNγ receptor 1 (**Fig 2f**)

When FRCs were separated from T cells and DCs by a semi-permeable membrane, the inhibitory effect was lost (**Fig 2g**). Addition of IFNγ itself also could not restore the inhibition in the transwell context, suggesting that a lack of IFNγ diffusion across the transwell didn't explain this effect. Combined with Fig 2e, this implied that, while IFNγ was involved, the inhibitory mechanism required cell-cell or very close proximity between T Cells, DC, and the modulating FRC population.

### Regulation of T cell priming by IFNγ-promoted Stromal iNOS

We therefore turned toward assessing mechanisms by which FRCs might inhibit T cell responses. Recent reports have shown that viral infection of FRCs results in their upregulation of PDL-1, an inhibitory molecule for T cells[12]. We assessed levels of PDL-1 as well as the costimulatory ligands CD86 (**Fig 3a**) and CD80 (data not shown). Whereas CD80 and CD86 levels were low and remained unchanged, PDL-1 levels were indeed upregulated in FRCs treated with IFNγ. However, blocking these pathways did not appreciably alter the proliferation of T cells in our assays (**Fig 3b**), suggesting another mechanism. Since IFNγ appeared to be necessary for inhibition, we next examined the transcription of *nos2* gene and protein expression and the production of nitric oxide (NO) which had previously been shown to be IFNγ-inducible in a selection of non-hematopoietic cells[15], [16] as well as cells of hematopoietic origin[17], [18]. The *nos2* gene encodes the enzyme inducible nitric oxide synthase (iNOS), which is responsible for production of nitric oxide and can be specifically inhibited by the drug 1400W. As shown in **Fig 3c**, addition of IFNγ directly to FRC lines in the absence of T cells or DCs results in an approximate 10-fold increase in transcription of the *nos2* gene, an effect that was not directly altered by blocking the enzyme itself with 1400W. Using antibodies to iNOS protein, we were able to detect significant signal by immunofluorescence in FRC lines and these levels were both quantitatively higher and more localized to the cytosol in the presence of T plus DC (**Fig 3d**, **arrowhead highlights T-DC couple**). Flow cytometry confirmed an upregulation of total iNOS levels in response to T+DC augmented, compared to control (DC alone), and that this augmentation could be blocked with antibodies to IFNγ (**Fig 3e**).

**Figure 3:** IFNγ dependent Induction of NOS2/iNOS/Nitrate production in Lymphoid stromal cells. (**a**) Costimulatory marker expression on the surface of FRC.5 cells following IFN**γ** treatment. (**b**) CFSE dilution profiles of OTI T cells stimulated with peptide-loaded BMDCs in the presence or absence of FRC.5 cells and blocking antibodies to CD80, CD86, or PDL-1. (**c**) Real-time PCR expression of *nos2* mRNA in FRC.5 cells cultured with either IFN**γ**, an iNOS-specific enzyme inhibitor (1400W), or both. (**d**) Immunofluorescence staining of NOS2 protein in FRC.5 cells cultured with pre-labeled SL8-pulsed BMDC or in the presence of pre-labeled SL8-pulsed BMDC plus pre-labeled T cells. Teal lines around FRC in FRC/DC condition indicate the border of the FRC and white arrowhead indicates a T-DC couple. Scalebar 20 µm. (**e**) Intracellular flow cytometry for NOS2 protein expression by FRC.5 cells cultured with SL8-pulsed BMDC with or without T cells and with or without IFN**γ** blockade for 48 hours. (**f**) Extracellular nitrite concentration measured by Griess assay in FRC.5 cultures either alone; with OTI T cells and peptide-loaded BMDCs; or OTI cells, peptide-loaded BMDCs, and 1400W.

We next measured accumulation of nitrite, a relatively-stable end-product of nitric oxide, in our cultures using a standard Griess assay[19]. Here, we found that addition of exogenous IFNγ to FRC cultures failed to increase production of nitrite to detectable levels (**Fig 3f**), an effect that may suggest that release or further activation of the enzyme requires additional signals delivered with T cell activation. However, nitrite was detected when T cells were stimulated in those cultures using SL8-loaded BMDCs, and this was considerably augmented by inclusion of FRC in a concentration-dependent manner. Nitrite could not be detected when unstimulated FRCs were plated. Finally, the nitrite that was detected when FRCs were mixed with T cells plus peptide-loaded DCs was blocked by the iNOS-specific inhibitor 1400W.

To test the emerging hypothesis that iNOS production was responsible for FRC inhibition of T cell responses, we mixed T cells plus SL8-loaded DCs together with FRCs in the presence or absence of iNOS inhibition. As shown in **Fig 4a**, we could completely restore proliferation of OTI CD8+ T cells by blocking iNOS function with 1400W. Similarly, we could restore proliferation using the drug L-NMMA, a broader-spectrum NOS inhibitor. When quantified as % blasts, this drug completely released cells to proceed into cycle (**Fig 4b**–**c**) with only very modest inhibition of complete cycling of cells as assessed by CFSE peaks.

**Figure 4:** A proximal role for iNOS during T cell priming by Lymphoid Stroma. (**a**) Proliferation of OTI cells stimulated with peptide-loaded BMDCs in the presence or absence of FRC.5 cells and either a broad NOS inhibitor (L-NMMA) or the iNOS inhibitor,1400W. (**b**–**c**) Proliferation assays identical to that in (a) but measuring the effect of NOS inhibitors under various concentrations of FRC.5 cells. (**b**) % Blasts quantified, demonstrating FRC inhibition is reversible with iNOS blockade across a range of FRC concentration. (**d**) Proliferation of OTI cells stimulated with peptide-loaded iNOS-/- BMDCs with or without added FRC. All assays were repeated in a minimum of 2 trials, and typically 4–6 independent trials and all conditions were assayed in triplicate. Error bars represent SD. (**e**–**j**) C57/Bl6 or *iNOS^−/−^* mice were immunized subcutaneously with either SL8 peptide-loaded BMDCs (**e**–**g**) or anti-DEC205-OVA conjugates (**h**–**j**) as described in Methods. Inguinal lymph nodes were isolated 3 days post-immunization, stained and analyzed by flow cytometry. (**e,h**) Relative recovery of total CD8^+^ cells in the inguinal lymph nodes of C57/Bl6 (n = 4) immunized mice relative to immunized *iNOS^−/−^* mice (n = 4). (**f,i**) The percentage of tetramer positive cells in the CD8^+^ compartment post-immunization. (**g,j**) The number of tetramer positive cells in immunized C57/Bl6 and *iNOS^−/−^* mice.

As iNOS has clearly been described as being produced by a variety of macrophages[17], [18], we wished to formally exclude that our BMDC were not in some way responsible for the production and inhibition. This was previously supported by our demonstration that FRC inhibited responses to anti-CD3 plus anti-CD28 or PMA/Ionomycin (Fig 1) and also the demonstration that 1400W augmented responses in the presence of FRC, but had no effect on basal proliferation in their absence (Fig 4b–c). Consistent with this, the stimulation of T cells using BMDC from mice genetically lacking the iNOS gene was nevertheless dramatically inhibited by stromal lines (**Fig 4d**). We noted that T cell inhibition by LEC or BEC stroma appears to operate via a similar iNOS/IFNγ dependent mechanism (data not shown).

Although it is currently not possible to generate a mouse in which deletion of iNOS is restricted to stroma and bone-marrow chimeras to approximate this fail to fully reconstitute the lymphoid compartment for unknown reasons (data not shown), we nevertheless sought to determine whether our findings were consistent with iNOS acting to attenuate T cell responses in lymph nodes. This was particularly important since previous reports had noted a requirement for iNOS in augmenting immune responses, likely as a result of its potent anti-microbial activity[20]–[22]. We therefore turned to the use of a germline *nos2* (iNOS) knockout and immunized in ways that should engage the pathway we had studied in vitro and, conversely, in ways that might not engage this mechanism. We additionally chose to use tetramer staining to examine the response derived from endogenous repertoire rather than using a TCR-transgenic adoptive transfer system that may bias the outcome due to abnormally high numbers of antigen-responsive cells.

To recapitulate our in vitro studies in which BMDC prime IFNγ production and the ensuing iNOS production, we first immunized control or iNOS^−/−^ mice in the flank using the same BMDCs pulsed with SL8 peptide. In this regimen, BMDC were always iNOS proficient and so any change due to the genetic background of the host would be due host cells beyond the APC. As shown in **Fig 4e**–**g** iNOS deficiency resulted in an overall trend towards an increased percentage of tetramer+ cells among total CD8 T cells and a statistically significant increase (1.8 fold) in the absolute number of tetramer+ CD8+ T cells in the lymph node at day 3.

As a comparison, we repeated this type of experiment but sought to direct antigens to a resident DC population in the absence of additional overt inflammatory cues. For this, we targeted the relatively non-inflammatory DEC-205+/CD8+ DC subset as antigen presenting cells[23] using anti-DEC205-OVA antibody-protein conjugates[24]. In contrast to what was observed using inflammatory DCs as the priming antigen presenting cells, iNOS deficiency consistently resulted in a mild decrease in T cell expansion as assessed using tetramer staining (**Fig 4h**–**j**). Together this suggests that iNOS production during intra- lymph node priming in the first 3 days does represent a mechanism of regulating T cell responses, as predicted by our *in vitro* experiments. Interestingly, and subject to further study, it also indicates that iNOS is differentially engaged and utilized, depending on the type of challenge and we would propose that this may depend upon the cell types that are stimulated to produce it and the local responses to this. The engagement of this pathway during the first days of lymph node priming will represent fruitful future study to understand the likely multiplicity of its action.

### FRC inhibition depends on T cell production of IFNγ and is Th1 specific

A key prediction of these results is that T cells that do not make IFNγ will not engage this regulatory mechanism. To formally test this, we assessed FRC-mediated inhibition of OTI cells lacking the interferon gamma gene (IFNγ−/−). As shown in **Fig 5a**, OTI T cells lacking expression of IFNγ were completely refractory to FRC-mediated inhibition, even when they were present at fractions as high as 10% of T cells. Confirming that this was truly due to the loss only of IFNγ, addition of exogenous IFNγ to these cultures re-established inhibition of T cell cycling.

**Figure 5:** FRC-mediated inhibition of IFNγ producing CD4+ and CD8+ T cells but not Th2 cells. (**a**) Percentage of blasting IFN**γ** ^−/−^OTI T cells cultured with peptide-loaded BMDCs and various concentrations of FRC.5 cells with or without exogenous IFN**γ**. (**b**) Dilution profiles of SE-eFluor670-labeled Th1 or Th2 skewed OTII cells when cultured with peptide-bearing BMDCs in the presence or absence of FRC.5 cells. (**c**) Quantification of SE-eFluor670 MFI (from (b)) as an index of proliferation (higher MFI represents reduced proliferation.) All experiments are representative of 2 similar trials. All conditions were assayed in triplicate.

This observation raised the possibility that FRCs might specifically block certain types of T cells that make IFNγ while sparing those that do not. A classic dichotomy exists in CD4 T cell subsets in which effector T helper 1 (Th1) cells produce IFNγ but no IL-4, whereas T helper 2 (Th2) cells produce IL-4 but no IFNγ. We therefore tested the prediction that FRCs would specifically block cycling of restimulated Th1 clones while having little or no effect on Th2 cells. As shown in **Fig 5b**–**c**, we found this to be the case: Th1 cells loaded with SE-efluor670 dye had a significantly higher MFI, indicative of less dilution and hence fewer rounds of cell division, when cultured with FRCs whereas Th2 cells showed no difference in MFI. Since blasts are heterogeneous in size and proliferate quickly from the start of this assay, we do not observe cells expressing undiluted levels of this dye. For this reason we did not quantify %Blasts for this assay. **Figure 5c** demonstrates that Th2 cells are insensitive to FRCs across a broad range of concentrations while Th1 cells proliferate less (higher SE-efluor670 MFI) as FRCs are added in increasing concentrations.

### FRCs block cell-cycle progression but do not block initial TCR recognition

We next turned toward dissecting the dynamics of how iNOS functions during the priming response. We first assessed the ability of T cells to form stable conjugates with DCs over time and found no significant difference between T cells activated with BMDCs in the presence of upwards of 25% FRCs (**Fig 6a**). Similarly, analysis of calcium signaling profiles failed to detect significant differences in the kinetics of intracellular calcium rise over the first 12 minutes post BMDC contact, despite the readily available co-engagement of these cells (**Fig 6b**). When examining the dynamics of the priming reaction, the first sign of inhibition by FRCs occurred at approximately 24 hours when cultures were examined for homotypic T-T clusters, correlating with successful activation[25], [26]. This timeframe has previously been shown to correspond to early IFNγ production in T cells[27]. OTI T cells cultured with SIINFEKL-pulsed DCs in the absence of FRCs displayed robust clusters averaging 1.2×10^4^ µm^2^ in size while average cluster size in the presence of FRC was 0.1×10^4^ µm^2^ (**Fig 6c**–**d**). This was, in part, mediated by the action of iNOS/NO production as homotypic clustering was partially restored by blockade with 1400W to an average size of 0.5×10^4^ µm^2^. The remaining inhibition may suggest a second mechanism that alters homotypic adhesiveness although this will be subject of future work.

**Figure 6:** Inhibition of T cell activation by LN stromal lines occurs largely at the level of cell-cycle progression. (**a**) Percentage of coupled OTI T cells and peptide-loaded BMDCs in the presence of various concentrations of FRC.5 cells. Cultures were analyzed at the times indicated post addition of OTIs. (**b**) Ratiometric measurement of cytosolic Ca^2+^ flux in FURA-2AM loaded OTI T cells, immediately after contact with peptide-bearing BMDCs in the presence or absence of FRC.5 cells. (**c**) Analysis of OTI and BMDC cluster area in the presence or absence of FRC.5 cells and iNOS inhibitor (1400W). (**d**) Images of T cell clusters under the conditions described in (**c**). Scale bar represents 100 um. (**c**,**d**) Cultures were incubated for 48 hours prior to imaging analysis. (**e**) Surface staining of OTI T cells for activation markers CD25 and CD69 after 24 hours when cultured with peptide-loaded BMDCs in the presence or absence of FRC.5 cells. Stains are compared to non-activated, naïve OTI T cells. (**f**) Percent of OTI cells with upregulated CD25 and CD69 levels following culture with BMDCs and various concentrations of FRC.5 cells for 36 hours. (**g**) Propidium iodide (PI) incorporation and Ki67 levels in OTI T cells at 36 hours under identical culture conditions as those in (**e**). (**h**–**i**) PI incorporation and Ki67 levels in OTI cells with various concentrations of FRC.5 cells. All experiments are representative of a minimum of 3 similar trials.

Interestingly, when we assessed CD25 and CD69 expression, markers of early T cell activation, we found only a small difference in CD25 upregulation at 24h when FRCs were added and no difference in CD69 upregulation at this time, regardless of how many FRC were in the culture (**Fig 6e**–**f**). In comparison, however, when cells were assessed at 36 hours for cell-cycle progression and the expression of Ki67, a marker of cell cycling, the profiles of T cells activated in the presence of FRC were identical to those of naïve T cells, showing very significant inhibition of these measures. This effect was titratable: between 1 and 2.5% FRCs, both progression to G2/M and the expression of Ki67 were reduced (**Fig 6g**–**i**). From this we conclude that the interactions occurring after initial T-DC interaction, but prior to approximately 36 hours, lead to the predominant inhibition of T cell proliferation. From our other evidence, this is consistent with published reports that OTI T cells generate IFNγ within the first 24 hours[27] and (our data) that T cell IFNγ production leads to FRC expression of iNOS in a similar timeframe. Consistent with our previous data, inhibition of NO production reverses the block in cell-cycle and overall expansion of the T cells (**Fig 6h**–**i** **)**

## Discussion

A key finding of this study is that FRCs are inhibitory to T cell responses. This inhibition of cell-cycle progression clearly depends upon a number of features of the priming reactions. First, FRCs sense early IFNγ. Thus, T cells that do not produce extensive cytokines of this class are less restricted. It is interesting, therefore, to note that Th2 cells are completely uninhibited by these effects. This may provide a basal bias towards non-inflammatory Th2 signaling, as T cells making these cytokines might be less likely to provoke inhibitory signaling from stromal sources. Speculatively, it may be that greater selective pressure exists to restrain local Th1-type responses given their ability to directly damage surrounding cells. In contrast, while grossly unrestrained Th2-responses are clearly detrimental, local controlled responses are more commonly associated with damage repair and tissue-beneficial roles. To this extent, the most important role of this mechanism might be tissue self-preservation in addition to T cell ‘tolerance’.

How inhibitory are FRCs in situ? In our in vitro experiments, we observed inhibition with as few as 1% FRCs relative to T cells. A conservative estimate is that FRCs are on the order of 50–100 times more sparse than T cells on a per-cell basis, and thus our assays are likely in the physiological range of cell number. In vivo, however, effects are almost certainly local. NO itself will not persist in interstitial spaces, largely because it nitrosylates proteins locally and is thereby consumed. Thus, under typical priming situations, there is unlikely to be ‘inhibition at a distance’. Rather only those T cells that remain in contact with iNOS producing cells will be inhibited in this way. This prediction is borne out in our transwell experiments (**Fig 2g**), which show that inhibition is essentially undetectable when cells are across the barrier, although there are detectable levels of NO in supernatants (**Fig 3f**). One prediction of this finding is that T cell responses that lead to extensive local ‘stopping’ of motile T cells within regions of the lymph nodes would be more susceptible to this cross-talk as compared to more transient and dynamic priming reactions. As clear modulation of this remains difficult, we are presently unable to directly test this prediction but the concept may force a re-evaluation of whether it will always be beneficial for T cells to stably reside at a single site in the lymph node, particular when IFNγ is elicited.

A related and important feature of this mechanism is that it is likely to not only be spatial, due to the short-range action of NO, but also to be temporal due to a specific window of IFNγ production and then a lag until FRCs respond by making iNOS. Bousso et. al recently showed that activated CD8 T cells produce IFNγ within 24-hours[27], thus providing a mechanism for our early IFNγ-iNOS axis. However, more typically, this cytokine may peak many hours or even days later. This delay may account for inhibition at 3+ days in vivo. In our hands, the method of priming even for immunization regiments altered the magnitude by which lymph node iNOS production affects priming. To this extent, FRCs may be induced to fully produce iNOS in some very late-stage responses and, given our finding that blasts can be inhibited and that inhibition of naïve cells occurs via late blocks in cell-cycle progression, T cells may also be similarly inhibited by stroma in these responses.

While FRCs are inhibitory, they are not alone in this capacity. As shown in **Figure 1e**, it is likely that many cell types, when added to T+DC priming reactions, may be inhibitory. This may be due to a selection of inhibitory factors or simply nutrient deprivation. However, the addition of IFNγ blocking antibodies in the FRC culture shows that the mechanisms by which FRCs attenuate T cell responses are not ‘non-specific’ but rely on direct sensing of the response. In that regard, too, iNOS responses like the ones discussed here have been previously reported in macrophages[17] as well as mesenchymal stem cells [15] and many other tissue stroma cells (e.g. in an accompanying paper by Luther et al.) A key distinction between our studies and those formerly mentioned is that we are now demonstrating this pathway to be actively engaged during specific types of T cell priming directly in the lymph node and via the lymph node structural cells, suggesting a more integral role, in the latter, in guiding the activation dynamics of Type 1-immune responses.

Is iNOS production by stromal cells always inhibitory to T cell function? Our data using direct targeting to DEC-205 antigen presenting cells indicates it most certainly will not be for all types of priming in the T cell compartment. And, from the global immune response, there are many reasons an ongoing immune response benefits from iNOS production. Most prominently, iNOS is upregulated in neutrophils in response to bacteria[28], is critical for resistance to Leishmania[20], and Listeria infection[21]. In this context, iNOS may lead to increased antigen presentation and improved overall outcome. However and notably, these mice have previously been shown to exhibit enhanced Th1 responses, a result which now may be partly or fully explained by the mechanism we describe here. The role of iNOS in the immune response therefore continues to evolve and may play positive and negative regulatory roles when expressed in stromal cells.

## Methods

### Mice

Ovalbumin-specific TCR transgenic OTI, OTII, OTI GFP and OTI IFNγ −/− mice were bred in-house. iNOS−/− mice[22] were gifts from L. Liu (University of California San Francisco) or purchased from the Jackson Laboratory (B6.129P2-*Nos2^tm1Lau^*/J). C57/Bl6 mice were purchased from the Simonsen Laboratory. All mice were maintained under specific pathogen-free conditions at the University of California San Francisco Animal Barrier Facility. Experimental procedures were approved by the Institutional Animal Care and Use Committee of the University of California San Francisco under protocol authorization number AN081824-03B.

### Antibodies, reagents, and flow cytometry

#### Flow Cytometry and Cell Sorting

αCD31(clone 390), αgp38(clone 8.1.1), αCD45(clone 30-F11), αCD25(clone PC61), αCD69(clone H1.2F3) and αCD8(clone 53-6.7) were purchased from BioLegend. αCD86(clone B7-2) and αCD279/PD1(clone J43) were purchased from eBioscience. αKi67(clone B56), αCD19(clone 1D3), αNOS2(anti-iNOS/NOS type II, polyclonal) and αIFNγR alpha chain(clone GR20) were purchased from BD. Tetramers specific for SIINFEKL peptide (SL8) bound to H-2K^b^ were purchased from ProImmune. For flow cytometry, cells were first blocked with αCD16/32 (clone 2.4G2) and then stained in PBS + 10% FCS with the antibodies listed above. For Intracellular staining of NOS2, cells were surface stained as described above (FACS only) and subsequently fixed 4% paraformaldehyde and then permeablized in PBS +10%FCS+0.5% Saponin: staining with αNOS2-FITC was then performed in this same permeabilization buffer at 4°C. Data was collected on either an LSRFortessa or a FACScalibur (BD) and analyzed using Flowjo (Treestar).

#### *In vitro* and *in vivo* T cell activation

αCD3(clone 2C11, produced in-house), αCD28(clone PV-1, University of California San Francisco Hybridoma Core Facility, UCSF-HCF), SL8 peptide (Anaspec),Ovalbumin peptide (323-339) (Genscript) PMA and ionomycin (Sigma-Aldrich). αCD40 (ebioscience), and IFNγ (Peprotech.) αDEC205-OVA (DEC-OVA) conjugates were produced in-house, using established protocols^3^.

#### In vitro blocking

Antibodies against IFNγ(clone XMG1.2, BioXCell), IL2(clone JES6-1A12, ebioscience) and PD1(clone RMP1-14, Biolegend). Antibodies against CD80(16-10A1) and CD86(GL-1) were purchased from UCSF-HCF.

#### Cytokine Stimulation and inhibitors

1400W and L-NG-monomethyl Arginine citrate (L-NMMA) were purchased from Sigma-Aldrich. IFNγ, IL4 and IL2 were purchased from Peprotech. IL2 was also produced in-house from transfected lines. The cellular dyes propidium iodide, CFSE, DDAO and FURA-2 AM were purchased from Invitrogen. Proliferation dye eFluor670 was purchased from eBioscience.

### Cell isolation

OTI T cells were isolated from the lymph nodes and spleen of 6 to 8 week old OTI mice. Selection was carried out using a negative CD8 isolation kit (STEMCELL Technologies Inc.). Cells were cultured in RPMI supplemented with 1 mM L-glutamine, penicillin, streptomycin, 5×10^−5^ M βME, and 10% FCS (R10). Th1 and Th2 cells were produced by isolating the spleen of OTII TCR transgenic mice and culturing 2×10^6^ cells with the following combination of reagents. Anti-CD28, anti-IL4, IL12, IL2 and Ovalbumin peptide (323–339) were added to produce Th1 cells. Anti-CD28, anti-IFNγ, IL4, IL2 and Ovalbumin peptide (323–339) were added to produce Th2 cells. Bone marrow-derived dendritic cells (BMDCs) were generated by culturing bone marrow cells for 7–10 days with GM-CSF in IMDM supplemented with 1 mM l-glutamine, penicillin, streptomycin, 5×10^−5^ M βME, and 10% FCS. IL4 was added for the last 2 days of culture.

### Generation of stromal cell lines

Peripheral lymph nodes from C57/Bl6 mice were isolated and ground between two microscope slides. Lymph node tissue was then digested for 20 minutes at 37°C in 2 ml of RPMI 1640 medium containing 2% FCS, collagenase IV (2 mg/ml; Sigma-Aldrich) and DNAseI (40 ug/ml; Roche). The tissue was then washed and resuspended in RPMI 1640 containing 2% FCS, collagenase D (1 mg/ml; Roche) and DNAseI (40 ug/ml) for further digestion. Throughout the digestion procedure fragments were gently sheared by passing through a 21.5 gauge needle every 10 minutes. When no visible fragments remained the sample was washed in RPMI 1640 medium containing 5 mM EDTA and finally resuspended in PBS containing 10% FCS at a concentration of 2×10^6^/ml. The resulting cell suspension was incubated at room temperature with 0.1 µg of 2.4G2 for 15 minutes. Without washing αCD31, αgp38, αCD45, and 1 µg DAPI were added to cells and incubated for an additional 30 minutes. Cells were then washed in sterile PBS + 10% FCS and sorted using a BD Biosciences FACSAria II Cell Sorter. Stromal populations were defined as FRC (FRC.5) CD31(−) gp38(+), LEC (LEC.6) CD31(+)gp38(+), and BEC (BEC.7) CD31(+) gp38(−) and sorted in sterile RPMI 1640 containing 50% FCS and subsequently washed and plated in sterile R10 media.

### RNA isolation and RT-PCR

RNA was extracted using the RNeasy Mini Kit from Qiagen. First strand synthesis was completed using random hexamers and reagents from the SuperScript III kit purchased from Invitrogen. 100 ng of cDNA was amplified using a SYBR Green PCR Master kit (Applied Biosystems) on a CFX96 real-time thermal cycler (Bio-Rad). Expression of *nos2* transcript is quantified as the amount relative to the expression of the housekeeping gene hypoxanthine guanine phosphoribosyl transferase (*Hprt1*). This measure is calculated with the following formula: 2^Ct(*Hprt1*)-Ct(*nos2*)^ where Ct(*Hprt1*) and Ct(*nos2*) represent the cycle number where the signal is amplified to a threshold value that is held constant between experiments. *nos2* transcript was amplified using the following primer sequences: ctcactgggacagcacagaa and gcttgtctctgggtcctctg (Integrated DNA Technologies).

### Proliferation assay

FRC.5 cells were plated at the amounts indicated, where ‘% of FRC’ refers to the percentage of FRC.5 cells relative to the total T cells in culture, in wells of a 96 well culture-treated dish 6 to 8 hours prior to the addition of T cells. OTI-GFP, Th1, Th2 and OTI-IFNγ^−/−^ T cells were purified as described above and labeled with either 2 µM CFSE or 4 µM eFluor670 proliferation dyes. 1×10^5^ T cells were added to FRC.5 cultures. Where indicated, T cells were activated with peptide-loaded BMDCs (1×10^4^ per well), plate-bound αCD3 (2 µg/ml), plate-bound αCD3 (2 µg/ml) and soluble αCD28 (2 µg/ml), or PMA (2 ng/ml) and ionomycin (20 ng/ml). BMDCs were matured with 1 µg/ml LPS 1 day before addition to cultures and pulsed with SL8 peptide (100 ng/ml) or Ovalbumin peptide 323–339 (250 ng/ml) for 1 hour. αCD3 was plated 16 to 24 hours prior to the addition of FRC.5 cells. Where indicated, T cell proliferation was augmented with the addition of various drugs, cytokines and antibodies at the start of the assay. Cultures were stained or fixed at the times noted and analyzed by flow cytometry.

### T-DC coupling assay

For *in vitro* T-DC coupling, BMDCs were matured with LPS (1 µg/ml) 1 day before priming and pulsed with SL8 peptide (100 ng/ml) for 1 hour. BMDCs and naïve OTI cells were labeled with 4 µM DDAO and 4 µM eFluor670, respectively. OTI cells were mixed with BMDCs at a ratio of T-DC 2:1. FRC.5 cells were added in the amounts indicated and the cell mixture was immediately centrifuged for 1 min at 228x*g* and incubated at 37°C. Cell mixtures were fixed at 15 minute intervals with an equal volume of warm 4% PFA in PBS. Cells were analyzed by flow cytometry for quantification of the percentage of couple formation, calculated as the number of T cells in the double-positive quadrant (eFluor670+ DDAO+) versus the total number of T cells (eFluor670+).

### Microscopy

The following techniques were used to image calcium flux in OTI T cells. Wells of a Lab-Tek II chambered coverglass system (Nunc) were plated with 7.5×10^4^ FRC.5 cells or fibronectin (1 µg/ml) 16 hours prior to the addition of BMDCs and OTI T cells. BMDCs were treated with LPS (1 µg/ml) 24 hours prior to the start of the assay and pulsed with SL8 peptide (100 ng/ml) for 1 hour. Naïve OTI-GFP cells were selected as described above and labeled with 4 µM FURA-2 AM for 45 minutes at 37°C. 7.5×10^4^ peptide-loaded BMDCs were added to wells containing FRC.5 cells or fibronectin coating 5 minutes before the addition of 2×10^5^ labeled naïve OTI cells. Interactions between BMDCs and OTI cells were visualized on a modified Zeiss Axiovert 200 M microscope with a 10x objective (Carl Zeiss). The microscope was fitted with dual excitation and emssion filter wheels, a Coolsnap-HQ camera (Photometrics) and a heated, motorized stage. Metamorph (Universal Imaging) was used as the imaging and control software. Data from DIC images, FURA emissions at 340 nm and 380 nm and green fluorescence were collected at 15-second intervals over a 20 to 30 minute period. Calcium flux was assessed based on the ratio of FURA-2 AM emissions at 340 nm to those at 380 nm, with increased ratios indicating calcium flux. Microscopy of NOS2 levels in mixed cultures utilized NOS2-FITC conjugates as described for FACS, utilizing cultures in which DC and/or T cells were separately pre-labeled prior to the initiation of cultures with FRC. Data was collected on a wide-field Zeiss 200 M microscope and analyzed in Metamorph.

The following techniques were used to image T cell clusters. 1×10^4^ FRC.5 cells or fibronectin were plated as described above. 6 hours later, 1×10^6^ naïve OTI-GFP cells and 1×10^5^ SL8 loaded BMDCs were added in the presence or absence of 1400W. Prior to imaging, chambers were spun down at 400x*g* for 1 minute. Images were captured on a modified Nikon Eclipse TE2000-S (Nikon). The microscope utilized a CSU10 confocal scanner unit (Yokagawa) and a XR Mega S-30 camera (Stanford Photonics). A custom build of Micromanager was used to control image acquisition. Data from DIC images and green fluorescence were collected. Cluster area measurements were conducted using the FIJI software suite of ImageJ.

### Measurement of NO production

Nitrite concentrations in culture supernatant were measured by the Griess assay as described previously[19]. Briefly, the culture supernatant was mixed sequentially with an equal volume of 1% sulfanilamide and 0.02% N-(1-naphthyl)ethylenediamine (0.5 M HCl) in a 96-well microplate. The absorbance at 540 nm was measured using a microplate reader, and the nitrite concentrations were derived from standard curves.

### Assessment of cell cycle status

Propidium iodide (PI) and Ki67 stains were performed on the proliferation assays described above. Cultures were spun down at 400x*g*, medium was aspirated and replaced with 70% ethanol for PI labeling or PBS containing 5% FCS and 0.5% saponin (Sigma-Aldrich) for Ki67 staining. Cultures were incubated for 1 hour in 70% ethanol prior to washing and subsequent PI staining (10 ug/ml in PBS containing 5% FCS). Percentage of cells actively cycling (in S, G2, or M phase) was calculated by taking the number of cells past the initial G_0_/G_1_ labeled peak and dividing by all live cells. Ki67 staining was performed immediately upon the addition of saponin medium. Cells were washed with PBS containing 10% FCS and analyzed by flow cytometry.

### Quantification of endogenous OVA-specific CD8 cells

Where indicated, mice were immunized with either BMDCs loaded with peptide or αDEC205-OVA conjugates. BMDCs were loaded with SL8 peptide (100 ng/ml) for 60 to 120 minutes at 37°C. Mice were immunized with a subcutaneous injection of 7.5×10^5^ BMDCs per flank in the presence of 200 ng/ml LPS in PBS. DEC205-OVA conjugates (3 µg) were administered subcutaneously in both flanks. At the times indicated, mice were euthanized and peripheral lymph nodes were excised. Lymph node cells were stained with R-PE conjugated MHC-I pentamer specific for the OVA peptide SIINFEKL in PBS containing 2% FCS. Subsequently, cells were stained for CD8 and CD19 and analyzed by flow cytometry.

## References

[1] Miller MJ, Safrina O, Parker I, Cahalan MD (2004). Imaging the single cell dynamics of CD4+ T cell activation by dendritic cells in lymph nodes.. J Exp Med.

[2] Mempel TR, Henrickson SE, Andrian von UH (2004). T-cell priming by dendritic cells in lymph nodes occurs in three distinct phases.. Nature.

[3] Hugues S, Fetler L, Bonifaz L, Helft J, Amblard F (2004). Distinct T cell dynamics in lymph nodes during the induction of tolerance and immunity.. Nat Immunol.

[4] Shakhar G, Lindquist RL, Skokos D, Dudziak D, Huang JH (2005). Stable T cell-dendritic cell interactions precede the development of both tolerance and immunity in vivo.. Nat Immunol.

[5] Stoll S, Delon J, Brotz TM, Germain RN (2002). Dynamic imaging of T cell-dendritic cell interactions in lymph nodes.. Science.

[6] Pflicke H, Sixt M (2009). Preformed portals facilitate dendritic cell entry into afferent lymphatic vessels.. J Exp Med.

[7] Gretz JE, Norbury CC, Anderson AO, Proudfoot AE, Shaw S (2000). Lymph-borne chemokines and other low molecular weight molecules reach high endothelial venules via specialized conduits while a functional barrier limits access to the lymphocyte microenvironments in lymph node cortex.. J Exp Med.

[8] Sixt M, Kanazawa N, Selg M, Samson T, Roos G (2005). The conduit system transports soluble antigens from the afferent lymph to resident dendritic cells in the T cell area of the lymph node.. Immunity.

[9] Bajénoff M, Egen JG, Koo LY, Laugier JP, Brau F (2006). Stromal cell networks regulate lymphocyte entry, migration, and territoriality in lymph nodes.. Immunity.

[10] Link A, Vogt TK, Favre S, Britschgi MR, Acha-Orbea H (2007). Fibroblastic reticular cells in lymph nodes regulate the homeostasis of naive T cells.. Nat Immunol.

[11] Mueller SN, Hosiawa-Meagher KA, Konieczny BT, Sullivan BM, Bachmann MF (2007). Regulation of homeostatic chemokine expression and cell trafficking during immune responses.. Science.

[12] Mueller SN, Matloubian M, Clemens DM, Sharpe AH, Freeman GJ (2007). Viral targeting of fibroblastic reticular cells contributes to immunosuppression and persistence during chronic infection.. Proc Natl Acad Sci USA.

[13] Constant S, Pfeiffer C, Woodard A, Pasqualini T, Bottomly K (1995). Extent of T cell receptor ligation can determine the functional differentiation of naive CD4+ T cells.. J Exp Med.

[14] Hosken NA, Shibuya K, Heath AW, Murphy KM, O'Garra A (1995). The effect of antigen dose on CD4+ T helper cell phenotype development in a T cell receptor-alpha beta-transgenic model.. J Exp Med.

[15] Sato K, Ozaki K, Oh I, Meguro A, Hatanaka K (2007). Nitric oxide plays a critical role in suppression of T-cell proliferation by mesenchymal stem cells.. Blood.

[16] Ren G, Zhang L, Zhao X, Xu G, Zhang Y (2008). Mesenchymal stem cell-mediated immunosuppression occurs via concerted action of chemokines and nitric oxide.. Cell Stem Cell.

[17] Albina JE, Abate JA, Henry WL (1991). Nitric oxide production is required for murine resident peritoneal macrophages to suppress mitogen-stimulated T cell proliferation. Role of IFN-gamma in the induction of the nitric oxide-synthesizing pathway.. J Immunol.

[18] Stuehr DJ, Nathan CF (1989). Nitric oxide. A macrophage product responsible for cytostasis and respiratory inhibition in tumor target cells.. J Exp Med.

[19] Eu JP, Liu L, Zeng M, Stamler JS (2000). An apoptotic model for nitrosative stress.. Biochemistry.

[20] Wei XQ, Charles IG, Smith A, Ure J, Feng GJ (1995). Altered immune responses in mice lacking inducible nitric oxide synthase.. Nature.

[21] MacMicking JD, Nathan C, Hom G, Chartrain N, Fletcher DS (1995). Altered responses to bacterial infection and endotoxic shock in mice lacking inducible nitric oxide synthase.. Cell.

[22] Laubach VE, Shesely EG, Smithies O, Sherman PA (1995). Mice lacking inducible nitric oxide synthase are not resistant to lipopolysaccharide-induced death.. Proc Natl Acad Sci USA.

[23] Winkel KD, Kronin V, Krummel MF, Shortman K (1997). The nature of the signals regulating CD8 T cell proliferative responses to CD8alpha+ or CD8alpha- dendritic cells.. Eur J Immunol.

[24] Hawiger D, Inaba K, Dorsett Y, Guo M, Mahnke K (2001). Dendritic cells induce peripheral T cell unresponsiveness under steady state conditions in vivo.. J Exp Med.

[25] Sabatos CA, Doh J, Chakravarti S, Friedman RS, Pandurangi PG (2008). A synaptic basis for paracrine interleukin-2 signaling during homotypic T cell interaction.. Immunity.

[26] Rothlein R, Springer TA (1986). The requirement for lymphocyte function-associated antigen 1 in homotypic leukocyte adhesion stimulated by phorbol ester.. J Exp Med.

[27] Beuneu H, Lemaître F, Deguine J, Moreau HD, Bouvier I (2010). Visualizing the functional diversification of CD8+ T cell responses in lymph nodes.. Immunity.

[28] Wheeler MA, Smith SD, García-Cardeña G, Nathan CF, Weiss RM (1997). Bacterial infection induces nitric oxide synthase in human neutrophils.. J Clin Invest.

